The article "Cerebral Venous Infarct After Recovery From COVID-19 Pneumonia" was retracted in 2024. Reasons: false authorship; unreliable results or conclusions; no approval from an author; concerns about the authorship.

# Cerebral Venous Infarct After Recovery From COVID-19 Pneumonia

**DOI:** 10.7759/cureus.19763

**Published:** 2021-11-20

**Authors:** Mohanned F Alfahhad, Saeed S Alghamdi, Osama A Alzahrani, Saleh K Aldakhil, Abdulaziz A Algarni, Ismail A Juraybi, Thekra M Alsalmi, Amjad S Alsulaihebi, Mawaddah K Yousef, Abdulaziz S Almuhaisen, Hamoud M Alfawzan, Fatema M Alsalehi, Raghad N Alsaeed, Hareth H Alharthi, Faisal Al-Hawaj

**Affiliations:** 1 College of Medicine, King Abdulaziz University, Jeddah, SAU; 2 College of Medicine, Al-Baha University, Al-Baha, SAU; 3 College of Medicine, Imam Mohammad Ibn Saud Islamic University, Riyadh, SAU; 4 College of Medicine, Jazan University, Jazan, SAU; 5 College of Medicine, Taif University, Taif, SAU; 6 College of Medicine, Umm Al-Qura University, Mecca, SAU; 7 College of Medicine, King Faisal University, Al-Ahsa, SAU; 8 College of Medicine, King Saud Bin Abdulaziz University For Health Sciences, Riyadh, SAU; 9 College of Medicine, Dammam Medical Complex, Dammam, SAU; 10 College of Medicine, Alfaisal University, Riyadh, SAU; 11 College of Medicine, Imam Abdulrahman Bin Faisal University, Dammam, SAU

**Keywords:** case report, computed tomography, cerebral venous sinus thrombosis (cvst), headache, coronavirus disease 2019 (covid-19)

## Abstract

The coronavirus disease 2019 (COVID-19) may have multisystem organ involvement. Thrombotic events are well-recognized complications of COVID-19. Such complications may include the pulmonary, renal, and other organs vasculature. The risk of coagulopathy is usually related to the severity of COVID-19 pneumonia. Few cases suggested that the coagulopathy risk may persist for some period after the recovery from COVID-19. We report the case of a middle-aged man with severe COVID-19 pneumonia that required seven days of endotracheal intubation and mechanical ventilation who presented with headache and left-sided weakness that occurred three days after his discharge. A computed tomography scan was performed to rule out intracranial hemorrhage before initiating the thrombolytic therapy. The scan demonstrated hemorrhage in the right temporal lobe with surrounding vasogenic edema along with density in the right transverse sinus. Subsequently, computed tomography venography was performed and demonstrated the filling defect representing right sigmoid venous sinus thrombosis. The patient received conservative measures in the form of intravenous hydration, anticoagulation, analgesics, and anticonvulsants. During the hospital stay, the patient had improvement in his symptom and mild neurological deficit persisted. The case highlighted that risk of thrombotic complications in COVID-19 pneumonia may persist for some period after the recovery from the disease. Hence, thromboprophylaxis may be indicated in selected patients with a risk of thrombotic events after their recovery from severe COVID-19.

The article "Cerebral Venous Infarct After Recovery From COVID-19 Pneumonia" was retracted in 2024. Reasons: false authorship; unreliable results or conclusions; no approval from an author; concerns about the authorship.

## Introduction

The coronavirus disease 2019 (COVID-19) is a primarily respiratory illness and has a wide range of multisystem complications. It became evident that thrombotic events are well-recognized complications of COVID-19 [1]. It has been reported that patients with COVID-19 may have coagulopathy with increased D-dimer levels. The thrombotic events may involve pulmonary, renal, and possibly cardiac vasculature [2]. Further, it was demonstrated that coagulopathy is directly related to the severity of COVID-19 [1]. However, few case reports highlighted the possible risk of coagulopathy even after the recovery from COVID-19. For example, Alqahtani et al. [3] reported a case of acute saddle aortic embolism that occurred three days after the recovery from severe COVID-19 pneumonia that required mechanical ventilation. Here, we report a similar case with a patient developing cerebral venous infarct following the recovery from severe COVID-19 pneumonia.

## Case presentation

We present the case of a 53-year-old man who was brought to the emergency department by ambulance because of severe shortness of breath. The patient developed shortness of breath seven days before his presentation and it was progressing in severity. The shortness of breath was associated with fever that reached 40℃ with a partial resolution with antipyretic medications. This was associated with a cough with purulent sputum. The patient had contact with a patient with COVID-19. However, he did not seek medical care. Further, the patient had previously refused to receive any vaccination for COVID-19. The past medical history was remarkable for severe gastroesophageal reflux disease for which he was taking oral omeprazole 40 mg for the last eight years. He underwent laparoscopic cholecystectomy as an elective operation after an episode of acute pancreatitis due to biliary stones. He was not known to have any drug or food allergies. He worked as an accountant and has a 35 pack-years history of smoking. He never consumed alcohol. The family history was remarkable for hereditary blood disorders, including glucose-6-phosphate dehydrogenase deficiency and beta-thalassemia.

Upon presentation, the patient appeared drowsy and was in respiratory distress. He was not able to speak in full sentences. He was using the accessory muscles of respiration. His vital signs showed tachycardia (120 bpm), tachypnea (25 bpm), fever (39.2℃), and maintained blood pressure (130/90 mmHg). His oxygen saturation was 79% on room air. Respiratory examination revealed decreased air entry with bilateral crepitations throughout both lung fields. Examination of other systems was unremarkable. Initial laboratory findings revealed a hemoglobin level of 13.1 g/dL, leukocytes count of 14,000/μL, platelets count of 410,000/μL. The inflammatory markers, including C-reactive protein (21.2 mg/dL) and the erythrocyte sedimentation rate (80 mm/hr), were elevated. Liver enzymes were mildly elevated with the level of alanine transferase level was 102 U/L and aspartate transferase was 58 U/L. Urea and electrolytes levels were within the normal reference range. Frontal chest x-ray revealed bilateral infiltrates suggestive of COVID-19. The diagnosis of COVID-19 was then confirmed by the reverse-transcriptase severe acute respiratory distress syndrome 2 (SARS-CoV-2).

The article "Cerebral Venous Infarct After Recovery From COVID-19 Pneumonia" was retracted in 2024. Reasons: false authorship; unreliable results or conclusions; no approval from an author; concerns about the authorship.

In view of the severe respiratory distress, the decision for endotracheal intubation and mechanical ventilation was made. The patient agreed to the plan. He was shifted to the intensive care unit and underwent intubation. Intravenous dexamethasone was administered. He received broad-spectrum antibiotic therapy in the form of ceftriaxone and gentamycin. Supplementary medications, including vitamin C and zinc, were given. The hemodynamic status of the patient was maintained and he did not require the use of inotropes. The patient developed gradual improvement in his condition and his oxygen requirement was decreasing. He was extubated after 8 days of intubation. He was weaned from supplementary oxygen gradually and his oxygen saturation was maintained on room air. He had a full recovery from the disease and was discharged after 14 days of hospitalization. He had no active complaints on the day of discharge.

Two days after discharge, the patient presented with severe headache and left-sided weakness that developed suddenly. Physical examination revealed left-sided weakness and slurred speech. The muscle power in the left upper limb was 3/5 and was 4/5 in the left lower limb. The fundoscopic examination was unremarkable for papilledema. The clinical picture was suggestive of an infarct in the territory of the left middle cerebral artery. Non-contrast computed tomography scan was performed to rule out any hemorrhage before initiating the thrombolytic therapy. The scan revealed a hemorrhage in the right temporal lobe with surrounding vasogenic edema. Further, a hyperdense right transverse sinus was noted (Figure 1). The scan was repeated after the administration of intravenous contrast and the images were acquired in the venous phase. The venogram confirmed the presence of right sigmoid sinus thrombosis by the presence of the filling defect (Figure 2).

The article "Cerebral Venous Infarct After Recovery From COVID-19 Pneumonia" was retracted in 2024. Reasons: false authorship; unreliable results or conclusions; no approval from an author; concerns about the authorship.

**Figure 1:** Non-contrast CT brain demonstrating right temporal lobe hemorrhage with a hyperdense right transverse sinus (arrow). CT: computed tomography

**Figure 2:** CT venography demonstrating a filling defect in the right sigmoid sinus (left circle) compared with the normal left sigmoid venous sinus (right circle). CT: computed tomography

Subsequently, the patient was managed conservatively and he did not develop neurological deterioration to necessitate surgical decompression. Fosphenytoin was administered as a prophylactic for seizures. Anticoagulant therapy was initiated despite the presence of intracranial hemorrhage. Parenteral analgesics in the form of non-steroidal inflammatory drugs relieved the patient’s headache. During the hospital stay, the patient had improvement in his symptom and mild neurological deficit persisted. He was discharged after one week of hospitalization. The patient underwent several physiotherapy sessions for his neurological deficit.

## Discussion

We reported a case of dural venous sinus thrombosis with cerebral hemorrhagic infarct in a patient recovering from COVID-19. Cerebral venous thrombosis is an uncommon type of stroke. It is three times more common among women [4]. Unlike other types of strokes, cerebral venous infarct often affects patients of younger ages. The pathogenesis of dural sinus thrombosis is incompletely understood. The most frequent risk factors include pregnancy, oral contraceptives, malignancy, infection, head trauma, and prothrombotic conditions [5]. In the present case, however, the patient did not have any of these factors.

Cerebral venous sinus thrombosis is a rare complication in COVID-19. In contrast to our case, the majority of reported cases of venous sinus thrombosis in the setting of COVID-19 were seen among women. The clinical manifestation is non-specific and includes a wide range of presentations. Cerebral venous sinus thrombosis may present with headache, fever, seizure, and altered level of consciousness [6].

While the coagulopathy risk was associated with the severity of COVID-19 [1], the risk of cerebral venous sinus thrombosis, in particular, does not seem to be directly related to the severity of COVID-19 [7]. The venous sinus thrombosis may develop even with mild symptoms of COVID-19 pneumonia [7]. As in the present case, intracranial hemorrhage is common after venous sinus thrombosis in COVID-19. For example, Abdelkader et al. [6] found that 25% of venous sinus thrombosis cases were complicated by cerebral venous hemorrhage.

Imaging studies are crucial to making the diagnosis of venous sinus thrombosis because of its non-specific clinical features. A computed tomography scan is often the first investigation performed in clinical practice. However, the scan may be normal in a significant number of patients [8]. Magnetic resonance imaging is the best imaging tool to confirm the diagnosis of venous sinus thrombosis, but it is not widely available. Hence, computed tomography venography is often the best alternative and it has a sensitivity of 95% [9].

The article "Cerebral Venous Infarct After Recovery From COVID-19 Pneumonia" was retracted in 2024. Reasons: false authorship; unreliable results or conclusions; no approval from an author; concerns about the authorship.

## Conclusions

Cerebral venous sinus thrombosis is a rare complication of COVID-19 pneumonia. The case highlighted that risk of thrombotic complications in COVID-19 pneumonia may persist for some period after the recovery from the disease. Hence, thromboprophylaxis may be indicated in selected patients with a risk of thrombotic events after their recovery from severe COVID-19. Since the radiological findings of venous sinus thrombosis may be subtle on computed tomography scan, a high index of suspicion is needed and computed tomography venography is the best alternative if magnetic resonance imaging is not available.
